The article "Protective Effects of Hydrogen on Myocardial Mitochondrial Functions in Septic Mice" was retracted in 2024. Reasons: signs of a paper mill; suspected computer-generated content; unreliable results or conclusions; concerns about the data.

# Protective Effects of Hydrogen on Myocardial Mitochondrial Functions in Septic Mice

**DOI:** 10.1155/2020/1568209

**Published:** 2020-01-30

**Authors:** Yuanyuan Zhang, Aili Dong, Keliang Xie, Yonghao Yu

**Affiliations:** Department of Anesthesiology, General Hospital of Tianjin Medical University, Tianjin, China

## Abstract

Enhancement of mitochondrial physiological function prevents sepsis-induced dysfunction. The present study aimed to elucidate the mechanism by which hydrogen (H_2_) affects mitochondrial function in a wild-type (WT) and homozygous nuclear factor erythroid 2-related factor 2 (Nrf2) knockout (KO, Nrf2^−/−^) murine model of sepsis. In myocardial tissues with severe sepsis, H_2_ gas treatment reduced mitochondrial dysfunction, whereas zinc protoporphyrin (ZnPPIX) negated these beneficial effects. H_2_ treatment upregulated the protein expression of mitofusin-2 (Mfn2), peroxisome proliferator-activated receptor-gamma coactivator-1*α* (PGC-1*α*), and protein heme oxygenase-1 (HO-1) in WT mice with severe sepsis but not in their Nrf2^−/−^ counterparts, and this upregulation was inhibited in the presence of ZnPPIX. In conclusion, the mechanism by which H_2_ limits organ damage in mice with severe sepsis involves HO-1, whereas the mechanism that limits severe sepsis-related mitochondrial dysfunction involves both HO-1 and Nrf2.

## 1. Introduction

Systemic inflammation in response to infection can lead to sepsis, which, when severe, is characterized by multiple-organ dysfunction syndrome [1]. In 2007 and 2013, 200,535 and 279,530 sepsis cases, respectively, were reported, indicating an annual rate of increase of 5.7% [2]. Despite a decrease in sepsis-related mortality in recent years, average associated mortality rates remain significant (e.g., 31.3% in the U.S. and 32.3% in Europe) [3].

The pathophysiology of sepsis and septic shock is strongly associated with the cardiovascular system, in which cardiac function plays a fundamental role. Animal-based studies of sepsis have identified mitochondrial dysfunction in a variety of tissues, such as the heart, skeletal muscles, and liver [4]. Cardiac myocytes play a central role in the pathogenesis of sepsis, as the ability of these cells to use oxygen during sepsis is compromised because of mitochondrial dysfunction, which leads to cellular energy depletion [5]. Previous studies have reported the role of various factors in cardiac injury during sepsis, and the protein heme oxygenase-1 (HO-1), a rate-limiting microsomal enzyme in the catabolism of heme into carbon monoxide, free iron, and biliverdin, limited septic injury by suppressing interleukin-1*β* and nuclear factor-*κ*B expression during the initial development of sepsis [6]. Furthermore, early inhibition of HO-1, also known as heat shock protein 32, during the development of an illness appeared to exacerbate septic damage. For example, treatment with zinc protoporphyrin IX (ZnPPIX) prior to cecal ligation and puncture (CLP) was associated with increased proinflammatory cytokine levels 6 h after the procedure [7]. In addition, nuclear factor erythroid 2-related factor 2 (Nrf2) is increasingly recognized as an important regulator of basal and induced expression of a range of antioxidant response element-dependent genes [8, 9]. Thus, Nrf2 regulates both physiological and pathophysiological responses to the presence of oxidants [10]. In the nucleus, the binding of Nrf2 to a DNA promoter under conditions of oxidative stress induced the transcription of antioxidant genes and subsequent translation of proteins, including HO-1 [11].

Hydrogen (H_2_) has been identified as a potential antioxidant in the context of both preventive and therapeutic approaches, given its antioxidant, anti-inflammatory, and antiapoptotic properties [12]. A compelling body of evidence supports the positive biological impacts of H_2_, which had positive therapeutic impacts in patients with more than 40 different illnesses and physiological conditions [13]. The fundamental mechanism underlying these positive effects has yet to be elucidated. A previous study found that H_2_ enhanced the expression and activity of HO-1 both *in vivo* and *in vitro* [14, 15]. Another study demonstrated that inhalation of 2% H_2_ could potentially alleviate intestinal damage caused by severe sepsis by regulating the release of HO-1 and high mobility group box 1 (HMGB1) [16]. Moreover, Nrf2 played a key role in the protective effect of H_2_ against intestinal injury [17].

Our previous investigations demonstrated increased survival and reduced injury and dysfunction in different organs (e.g., lungs, liver, kidney, and intestinal tract) in various septic models treated with H_2_ inhalation [17–19]. In the present study, using a CLP model, we investigated whether HO-1 mediated the positive effects of H_2_ on myocardial injury in a murine model of sepsis.

## 2. Materials and Methods

### 2.1. Experimental Design

This work used murine models approved by the Institute for Cancer Research. All experimental procedures were conducted after receiving approval from the Animal Experimental Ethics Committee of Tianjin Medical University General Hospital, Tianjin, China. Wild-type (WT) and Nrf2 knockout (KO) male mice (body weight: 20–25 g; age: 6–8 wk) were supplied by the Better Biotechnology Company (Nanjing, China). The mice were housed in cages (five mice per cage) in an environmentally controlled environment (temperature: 22–25°C) under an automated 12-h/12-h light/dark cycle, with food, and water *ad libitum*.

First, 16 WT and 16 Nrf2^−/−^ mice were arbitrarily divided into the following four groups, with eight mice in each group: (i) CLP, (ii) CLP + H_2_, (iii) KO + CLP, and (iv) KO + CLP + H_2_. Another 32 male WT mice were then arbitrarily divided into the following four groups (*n* = 8 in each): (i) CLP, (ii) CLP + H_2_, (iii) CLP + ZNPPIX, and (iv) CLP + ZNPPIX + H_2_. In both experiments, the mice were anaesthetized using 200 mg/kg of sodium pentobarbital 24 h after the commencement of CLP. Cardiac samples were collected from all mice.

CLP was used to induce sepsis according to previously described procedures [18]. ZNPPIX (40 mg/kg) was administered 1 h preoperatively via injection to mice in the CLP + ZNPPIX and CLP + ZNPPIX + H_2_ groups. Prior to the surgical procedure, the mice were anaesthetized using a 50 mg/kg dose of sodium pentobarbital (Sigma-Aldrich, St. Louis, MO, USA) administered by an intraperitoneal injection. Subsequently, a midline incision was made, and the cecum was exposed, ligated 1 cm from the apex, and punctured twice (through-through) using a 20-gauge needle. To ascertain the success of the punctures, a small quantity of fecal material was gently squeezed from the cecum. Subsequently, the cecum was relocated, and the peritoneum and skin were closed using 4/0 sutures. The control mice were subjected to a mock operation involving only incision and cecum externalization. Immediately following the procedure, all mice received 1 ml of a saline solution administered intravenously and were provided with a standard laboratory diet and drinking water *ad libitum*. Mice subjected to both the mock and CLP procedures were monitored for 7 d to evaluate survival.

All mice assigned to receive the H_2_ treatment were placed in a sealed plastic box fitted with inflow and outflow outlets [20]. These mice breathed a mixture of air and H_2_ gas supplied at a rate of 4 L/min by a TF-1 gas flowmeter (YUTAKA Engineering Corp, Tokyo, Japan). An HY-ALERTA handheld detector (Model 500; H_2_ Scan, Valencia, CA, USA) was used to continuously monitor the concentration of H_2_ in the box. The concentration was maintained at 2% during the treatment period. The mice inhaled 2% H_2_ for 60 min periods at the 1 h and 6 h time points after the CLP or mock procedure. The mice in the groups not treated with H_2_ breathed normal air.

### 2.2. Isolation of Mitochondria

Complete mitochondria were isolated from harvested cardiac tissue using the differential centrifugation procedure described by Drew and Leeuwenburgh [21]. A Potter–Elvehjem glass-glass homogenizer was used to homogenize the cardiac tissue in a 1 : 10 wt/vol mixture of ice-cold water and buffer A consisting of mannitol (0.220 M), sucrose (0.070 M), EGTA (0.5 mM), HEPES (2 mM, pH 7.4), and fatty acid-free bovine serum albumin (0.1%). Homogenates of cardiac tissues were then centrifuged at 1,600 *g* and 4°C for 10 min in an Eppendorf 5810R device (Brinkmann Instruments, Laurel, MD, USA). The supernatants were subsequently isolated and subjected to centrifugation at 18,000*g* and 4°C for 10 min, and the resultant pellets were resuspended in buffer A prior to an additional 10 min centrifugation step at 18,000*g* and 4°C.

Samples obtained from the frontal cortex of the brain were similarly homogenized in a 1 : 10 wt/vol mixture of ice water and buffer B, which consisted of HEPES-KOH (20 mM, pH 7.5), KCl (10 mM), MgCl_2_ (1.5 mM), EDTA (1 mM), EGTA (1 mM), DTT (1 mM), and PMSF (0.1 mM). After centrifugation of this homogenate at 750*g* and 4°C for 5 min, the supernatant was removed and subjected to centrifugation at 8,000*g* and 4°C for 20 min. After resuspending the pellets, the freshly separated mitochondria were immediately subjected to further analysis.

### 2.3. Measurements of the Mitochondrial Respiratory Control Ratio (RCR), Adenosine Triphosphate (ATP) Level, and Mitochondrial Membrane Potential (MMP)

The respiratory control ratio (RCR), a measure of the stability and energy-conserving capability of the mitochondrial membrane, was evaluated according to the method of Silva et al. [19] as the ratio between state 3 and state 4 respiration rates. The total cellular ATP level was assessed using an ATP bioluminescence assay kit according to the manufacturer's protocol (CLS II; Roche Applied Science, Mannheim, Germany). This protocol required collected cells to be counted using a Scepter cell counter (Millipore, Billerica, MA, USA). Subsequently, the cells were induced to release cellular ATP by adding the cell suspension to a boiling buffer consisting of Tris (100 mM) and EDTA (4 mM, pH 7.75) for 2 min. The bioluminescence signal was measured after diluting the reaction solution 1 : 1 (v/v) with luciferase reagent. ATP values were obtained by dividing the concentrations of ATP (determined using a standard curve) by the cell count [22]. The MMP was then assessed using an assay described by Sakamuru et al. [23].

### 2.4. Western Blotting

Twenty-four hours after both the CLP and mock operations, proteins were extracted from the harvested cardiac tissues and evaluated using a BCA protein assay kit (Pierce Biotechnology, Rockford, IL, US). Fifty-microgram aliquots of protein from each lysate were fractionated by 10% SDS-polyacrylamide gel electrophoresis and transferred to polyvinylidene difluoride membranes (Millipore, Billerica, MA, USA)), which were then blocked in a solution of 5% nonfat milk in phosphate-buffered saline-Tween-20 for 1 h at room temperature before blotting with the relevant primary antibody. Glyceraldehyde-3-phosphate dehydrogenase was detected as a loading control. The membranes were then washed four times with Tris-buffered saline and Tween-20, followed by incubation for 2 h with appropriate horseradish peroxidase-conjugated secondary antibodies (antirabbit or antimouse; Santa Cruz Biotechnology, Dallas, TX, USA). Quantity One software, version 4.5.2 (Bio-Rad, Hercules, CA, USA), was used to visualize the blots, and Gel-Pro analyzer (Media Cybernetics Inc., Rockville, MD, USA) was used to examine the integrated optical densities. For comparisons among experimental conditions, all changes in protein levels are presented relative to the control levels (i.e., the mock procedure).

### 2.5. Statistical Analysis

All statistical values are presented as means ± standard deviations. All analyses were performed using SPSS, version 20.0 (SPSS, Inc., Chicago, IL, USA). Differences between the mock procedure and CLP groups and those between the CLP + H_2_ and CLP groups were examined using an unpaired *t*-test. The Mann–Whitney *U* test was used for nonnormally distributed values. *P* values of <0.05 were considered statistically significant.

## 3. Results

### 3.1. Effect of H_2_ on Mitochondrial Physiological Function

To evaluate general mitochondrial function, we evaluated the RCR in the different groups of sepsis model mice. As shown in Figure 1, the RCR increased significantly in the CLP + H_2_ group relative to that in the other groups (*P* < 0.05) but decreased significantly in the KO + CLP group relative to that in the CLP group (*P* < 0.05). We detected no significant differences in the RCR in a comparison of the KO + CLP + H_2_ group with the CLP and KO + CLP groups (Figure 1(a)). Similarly, the ATP level (Figure 1(b)) and MMP (Figure 1(c)) increased significantly in the CLP + H_2_ group relative to that in the other three groups (*P* < 0.05) but decreased significantly when compared with that in the CLP group (*P* < 0.05). We detected no significant differences in the ATP level and MMP in the KO + CLP + H_2_ group compared with that in the CLP and KO + CLP groups.

When the mitochondrial status during the ZnPPIX treatment was evaluated, we observed the same trends in the RCR (Figure 2(a)), ATP level (Figure 2(b)), and MMP (Figure 2(c)) in the four groups. The RCR, ATP level, and MMP increased significantly in the CLP + H_2_ group when compared with that in the other three groups (*P* < 0.05), whereas no significant differences in these parameters were observed among the CLP, CLP + ZnPPIX, and CLP + ZnPPIX + H_2_ groups.

### 3.2. Effect of H_2_ on the Nrf2/HO-1 Pathway in WT and Nrf2^−/−^ Mice

We also measured the levels of several proteins. As shown in Figure 3, the levels of HO-1, mitofusin-2 (Mfn2), and peroxisome proliferator-activated receptor-gamma coactivator-1*α* (PGC-1*α*) increased significantly, and the level of dynamin-related protein 1 (Drp1) decreased significantly in the CLP + H_2_ group relative to that in the other three groups (*P* < 0.05). However, we detected no differences in the expression of HO-1, Mfn2, PGC-1*α*, and Drp1 among the CLP, KO + CLP, and KO + CLP + H_2_ groups.

Figure 4 shows the protein levels during the ZnPPIX treatment. The Drp1 level decreased significantly in the CLP + H_2_ group relative to that in the other three groups (*P* < 0.05) but increased significantly in the CLP + ZnPPIX and CLP + ZnPPIX + H_2_ groups as compared with that in the CLP group (*P* < 0.05). The CLP + H_2_ group had significantly higher levels of Mfn2, HO-1, and PGC-1*α* when compared with those in the other three groups (*P* < 0.05), whereas the levels of Mfn2 and HO-1 in the CLP + ZnPPIX and CLP + ZnPPIX + H_2_ groups were significantly lower than those in the CLP group (*P* < 0.05). Although the PGC-1*α* level in the CLP + ZnPPIX group was significantly lower than that in the CLP group (*P* < 0.05), no difference in the expression of this protein was observed in the CLP versus the CLP + ZnPPIX + H_2_ groups.

## 4. Discussion

The CLP procedure is a well-established, clinically germane method for generating models used in sepsis research [8, 9]. Mice with severe CLP-induced sepsis exhibit increased damage, compared with nonseptic mice. Previous research reported that inhalation of H_2_ gas at low concentrations (e.g., 2%) reduced the effects of sepsis and had therapeutic benefits in other illnesses [17]. In the present study, which included both WT and Nrf2^−/−^ mice, we demonstrated beneficial effects of inhaled H_2_ on mitochondrial function, as well as the central importance of Nrf2 and its downstream targets in this process.

Mitochondria are critical to the physiological processes of cells, and mitochondrial dysfunction has been linked to a wide range of illnesses, including cancer, cardiovascular diseases, diabetes, and neurodegenerative conditions [24–26]. The mitochondrion is often referred to as the powerhouse of the cell, as the eukaryotic cell derives almost its entire energy balance from oxidative phosphorylation in this organelle. Within the mitochondrion, electrons are transferred from electron donors to electron acceptors (e.g., oxygen) via a sequence of redox reactions along the electron transport chain. This transfer yields an electrochemical gradient that drives the synthesis of ATP and provides a central criterion for the assessment of the MMP, a marker of mitochondrial function [15, 27]. The actions of noxious xenobiotic substances can directly or indirectly affect mitochondrial function, and such substances often disrupt various mitochondrial macromolecules and thus reduce the MMP, which in turn compromises several mitochondrial functions [15, 27].

Defects in mitochondrial dynamics involve changes in mitochondrial fission/fusion proteins, such as Drp1 and mitofusins (e.g., Mfn2) [28]. These dynamic changes are regulated by complex mechanisms that maintain mitochondrial function homeostasis. Mitochondrial fission begins with the induction of Drp1. Mitochondrial fusion is a complex physiological process that involves optic atrophy 1 in the outer membrane and Mfn2 in the inner membrane [29] and depends on the MMP and hydrolysis of guanosine-5′-triphosphate [30]. The present investigation demonstrated reduced cardiac mitochondrial function in septic Nrf2^−/−^ mice as compared with that in their WT counterparts. Furthermore, the exacerbation of mitochondrial dysfunction observed in the Nrf2^−/−^ mice were accompanied by notable upregulation in Drp1 levels and considerable reductions in Mfn2 and PGC-1*α* levels relative to corresponding levels in the CLP group. The observed significant enhancing effect of H_2_ on mitochondrial function in septic mice involved Nrf2-mediated signaling in asepsis, as shown by the absence of any therapeutic benefit in the Nrf2^−/−^ mice.

The Nrf2 transcription factor is a central regulator of relevant innate immune responses and a mediator of antioxidant and anti-inflammatory responses [31]. This protein is transported from the cytoplasm into the nucleus, where it can bind to the (antioxidant responsive element (ARE) gene and thus regulate the expression and activation of antioxidants (e.g., Superoxide dismutase, catalase) and phase II genes (e.g., glutathione S-transferase, NAD (P)H quinine oxidoreductase, and HO-1) [32, 33]. The downstream enzyme HO-1 can break down the proinflammatory molecule heme to generate anti-inflammatory carbon monoxide and bilirubin, thus potentially moderating the inflammatory response [34]. Previously, our research group demonstrated a notable increase in the levels of Nrf2 and HO-1 in septic cell models and septic organs (lung, intestine, brain, and kidney) from mice in the presence of 0.6 mmol/L of H_2_-rich medium or the inhalation of 2% H_2_ [17].

Numerous *in vivo* and *ex vivo* experimental models have used ZnPPIX and other metallic morpholines as standard HO-1 inhibitors [35]. In the present study, ZnPPIX completely negated the beneficial effects of H_2_ treatment, including the observed increases in the RCR, MMP, ATP, and mitochondrial function-related protein expression. This finding further supports the ability of H_2_ to provide protection against sepsis by upregulating the expression of HO-1. In our study, the H_2_ treatment did not enhance the expression or activity of HO-1 or improve mitochondrial function and kinetics in the Nrf2^−/−^ mice. In addition, the use of ZnPPIX to inhibit HO-1 further demonstrated that the protective effects of H_2_ treatment for sepsis involved mitochondrial function and HO-1. Based on these findings, we conclude that H_2_ enhances mitochondrial performance by controlling mitochondrial activity via the Nrf2/HO-1 pathway.

In conclusion, the present investigation indicates the therapeutic potential of 2% H_2_ via inhalation for the management of mitochondrial dysfunction associated with severe sepsis. Furthermore, it suggests that these protective effects are mediated by a mechanism involving the regulation of HO-1 and Nrf2.

## Figures and Tables

**Figure 1:** Effects of H_2_ on mitochondrial function in a septic model of WT and Nrf2^−/−^ mice. RCR, respiratory control ratio; MMP, mitochondrial membrane potential. ^*∗*^*P* < 0.05 (*n* = 8).

**Figure 2:** Effects of H_2_ and ZnPPIX on mitochondrial function in a septic murine model. RCR, respiratory control ratio; MMP, mitochondrial membrane potential. ^*∗*^*P* < 0.05 (*n* = 8).

**Figure 3:** Effects of H_2_ on mitochondrial protein expression in heart tissue of WT and Nrf2^−/−^ mice. Mfn2, mitofusin-2; Drp1, dynamin-related protein 1; PGC-1*α*, peroxisome proliferator-activated receptor-gamma coactivator-1*α*; HO-1, heme oxygenase-1 HO-1. ^*∗*^*P* < 0.05 (*n* = 8).

**Figure 4:** Effects of H_2_ and ZnPPIX on mitochondrial protein expression in heart tissues. Mfn2, mitofusin-2; Drp1, dynamin-related protein 1; PGC-1*α*, peroxisome proliferator-activated receptor-gamma coactivator-1*α*; HO-1, heme oxygenase-1 (HO-1). ^*∗*^*P* < 0.05 (*n* = 8).

## Data Availability

All data are available at Dr. Yuanyuan Zhang yzhang10@tmu.edu upon request.

## References

[1] Iskander K. N., Osuchowski M. F., Stearns-Kurosawa D. J. (2013). Sepsis: multiple abnormalities, heterogeneous responses, and evolving understanding. *Physiological Reviews*.

[2] Fleischmann C., Thomas-Rueddel D. O., Hartmann M. (2016). Hospital incidence and mortality rates of sepsis. *Deutsches Aerzteblatt Online*.

[3] Levy M. M., Artigas A., Phillips G. S. (2012). Outcomes of the surviving sepsis campaign in intensive care units in the USA and Europe: a prospective cohort study. *The Lancet Infectious Diseases*.

[4] Zhang H., Liu D., Wang X. (2013). Melatonin improved rat cardiac mitochondria and survival rate in septic heart injury. *Journal of Pineal Research*.

[5] Landesberg G., Levin P. D., Gilon D. (2015). Myocardial dysfunction in severe sepsis and septic shock: no correlation with inflammatory cytokines in real-life clinical setting. *Chest*.

[6] Luo Y. P., Jiang L., Kang K. (2014). Hemin inhibits NLRP3 inflammasome activation in sepsis-induced acute lung injury, involving heme oxygenase-1. *International Immunopharmacology*.

[7] Kang K., Nan C., Fei D. (2013). Heme oxygenase 1 modulates thrombomodulin and endothelial protein C receptor levels to attenuate septic kidney injury. *Shock*.

[8] Calsavara A. C., Soriani F. M., Vieira L. Q., Costa P. A., Rachid M. A., Teixeira A. L. (2015). TNFR1 absence protects against memory deficit induced by sepsis possibly through over-expression of hippocampal BDNF. *Metabolic Brain Disease*.

[9] Zhang Y., Dong A., Xie K., Yu Y. (2019). Dietary supplementation with high fiber alleviates oxidative stress and inflammatory responses caused by severe sepsis in mice without altering microbiome diversity. *Frontiers in Physiology*.

[10] Ma Q. (2013). Role of Nrf2 in oxidative stress and toxicity. *Annual Review of Pharmacology and Toxicology*.

[11] Nguyen T., Nioi P., Pickett C. B. (2009). The Nrf2-antioxidant response element signaling pathway and its activation by oxidative stress. *Journal of Biological Chemistry*.

[12] Ohsawa I., Ishikawa M., Takahashi K. (2007). Hydrogen acts as a therapeutic antioxidant by selectively reducing cytotoxic oxygen radicals. *Nature Medicine*.

[13] Ohta S. (2014). Molecular hydrogen as a preventive and therapeutic medical gas: initiation, development and potential of hydrogen medicine. *Pharmacology & Therapeutics*.

[14] Chen H., Xie K., Han H. (2015). Molecular hydrogen protects mice against polymicrobial sepsis by ameliorating endothelial dysfunction via an Nrf2/HO-1 signaling pathway. *International Immunopharmacology*.

[15] Dong A., Yu Y., Wang Y. (2018). Protective effects of hydrogen gas against sepsis-induced acute lung injury via regulation of mitochondrial function and dynamics. *International Immunopharmacology*.

[16] Yu Y., Yang Y., Yang M., Wang C., Xie K., Yu Y. (2019). Hydrogen gas reduces HMGB1 release in lung tissues of septic mice in an Nrf2/HO-1-dependent pathway. *International Immunopharmacology*.

[17] Yu Y., Yang Y., Bian Y. (2017). Hydrogen gas protects against intestinal injury in wild type but not NRF2 knockout mice with severe sepsis by regulating HO-1 and HMGB1 release. *Shock*.

[18] Xie K., Yu Y., Pei Y. (2010). Protective effects of hydrogen gas on murine polymicrobial sepsis via reducing oxidative stress and HMGB1 release. *Shock*.

[19] Xie K., Yu Y., Huang Y. (2012). Molecular hydrogen ameliorates lipopolysaccharide-induced acute lung injury in mice through reducing inflammation and apoptosis. *Shock*.

[20] Li Y., Xie K., Chen H., Wang G., Yu Y. (2015). Hydrogen gas inhibits high-mobility group box 1 release in septic mice by upregulation of heme oxygenase 1. *Journal of Surgical Research*.

[21] Drew B., Leeuwenburgh C. (2003). Method for measuring ATP production in isolated mitochondria: ATP production in brain and liver mitochondria of fischer-344 rats with age and caloric restriction. *American Journal of Physiology-Regulatory Integrative and Comparative Physiology*.

[22] Liemburg-Apers D. C., Schirris T. J. J., Russel F. G. M., Willems P. H. G. M., Koopman W. J. H. (2015). Mitoenergetic dysfunction triggers a rapid compensatory increase in steady-state glucose flux. *Biophysical Journal*.

[23] Sakamuru S., Attene-Ramos M. S., Xia M. (2016). Mitochondrial membrane potential assay. *Methods in Molecular Biology*.

[24] Nicolson G. L. (2014). Mitochondrial dysfunction and chronic disease: treatment with natural supplements. *Alternative Therapies in Health and Medicine*.

[25] Wang D., Li S., Jiang J. (2019). Chinese society of cardiology expert consensus statement on the diagnosis and treatment of adult fulminant myocarditis. *Science China Life Sciences*.

[26] Zhang X., Liu H., Gao J. (2019). Metabolic disorder in the progression of heart failure. *Science China Life Sciences*.

[27] Schloesser A., Esatbeyoglu T., Piegholdt S. (2015). Dietary tocotrienol/gamma-cyclodextrin complex increases mitochondrial membrane potential and ATP concentrations in the brains of aged mice. *Oxidative Medicine and Cellular Longevity*.

[28] DuBoff B., Feany M., Götz J. (2013). Why size matters–balancing mitochondrial dynamics in Alzheimer’s disease. *Trends in Neurosciences*.

[29] Burté F., Carelli V., Chinnery P. F., Yu-Wai-Man P. (2015). Disturbed mitochondrial dynamics and neurodegenerative disorders. *Nature Reviews Neurology*.

[30] Beręsewicz M., Boratyńska-Jasińska A., Charzewski Ł. (2017). The effect of a novel c.820C > T (Arg274Trp) mutation in the mitofusin 2 gene on fibroblast metabolism and clinical manifestation in a patient. *PLoS One*.

[31] Vriend J., Reiter R. J. (2015). The Keap1-Nrf2-antioxidant response element pathway: a review of its regulation by melatonin and the proteasome. *Molecular and Cellular Endocrinology*.

[32] Liu G., Yu L., Fang J. (2017). Methionine restriction on oxidative stress and immune response in dss-induced colitis mice. *Oncotarget*.

[33] Xu K., Liu G., Fu C. (2018). The tryptophan pathway targeting antioxidant capacity in the placenta. *Oxidative Medicine and Cellular Longevity*.

[34] Vijayan V., Baumgart-Vogt E., Naidu S., Qian G. F., Immenschuh S. (2011). Bruton’s tyrosine kinase is required for TLR-dependent heme oxygenase-1 gene activation via Nrf2 in macrophages. *Journal of Immunology*.

[35] Hirai K., Sasahira T., Ohmori H., Fujii K., Kuniyasu H. (2007). Inhibition of heme oxygenase-1 by zinc protoporphyrin IX reduces tumor growth of LL/2 lung cancer in C57BL mice. *International Journal of Cancer*.

